# Prognosis Analysis and Perioperative Research of Elderly Patients with Non-Muscle-Invasive Bladder Cancer under Computed Tomography Image of Three-Dimensional Reconstruction Algorithm

**DOI:** 10.1155/2022/6168528

**Published:** 2022-06-06

**Authors:** Hongying Ke, Dandan Qiu, Zhicheng Cong

**Affiliations:** ^1^Department of Geriatrics, Zhejiang Hospital, Hangzhou 310000, Zhejiang, China; ^2^Department of Urology, The First Affiliated Hospital of Zhejiang Chinese Medical University, Hangzhou 310000, Zhejiang, China; ^3^Department of Urology, Zhejiang Hospital, Hangzhou 310000, Zhejiang, China

## Abstract

To analyze the application value of computed tomography (CT) based on a three-dimensional reconstruction algorithm in perioperative nursing research and prognosis analysis of non-muscle-invasive bladder cancer (NMIBC), a retrospective study was performed on 124 patients with NMIBC who underwent surgical treatment in the hospital. All patients underwent CT examination based on the three-dimensional reconstruction algorithm before surgery, and transurethral resection of the bladder tumor was performed. The patients receiving conventional care were classified as the control group, and those receiving comprehensive care were classified as the case group, and the recovery status and recurrence of the two groups were compared. The results showed that the accuracy, specificity, and sensitivity of CT imaging information based on the three-dimensional reconstruction algorithm for NMIBC patients were 89.38, 93.77, and 84.39, respectively. The incidence of bladder spasm (9.68%), bladder flushing time (1.56 d), and retention of drainage tube time (2.68 d) in the case group were obviously lower compared with the control group (30.65%, 2.32 d, and 5.19 d) (*P* < 0.05). Serum BLCA-1 (3.72 ng/mL) and CYFRA21-1 (5.68 *μ*g/mL) in the case group were significantly lower than those in the control group, with a statistically considerable difference (*P* < 0.05). Compared with the control group, the scores of role function (89.82 points), emotional function (84.76 points), somatic function (79.23 points), and social function (73.93 points) in the case group were observably higher (*P* < 0.05). In addition, one year after the operation, CT examination showed that the recurrence rate in the case group (6.45%) was significantly lower than that in the control group (22.58%) (*P* < 0.05). Therefore, CT detection based on the three-dimensional reconstruction algorithm was particularly important for preoperative diagnosis, prognosis, and recurrence monitoring of NMIBC patients. It could provide great clinical value for the diagnosis and prognosis monitoring of NMIBC.

## 1. Introduction

In recent years, the incidence rate of bladder cancer has been increasing. As the most common malignant tumor of the urinary system, it brought great threat and harm to patients both at home and abroad [1, 2]. North America, North Africa, and Europe are the most frequent areas of bladder cancer worldwide. Egypt has the highest incidence rate of cancer in the world. In addition, statistics showed that in 2010, the number of new bladder cancer patients in the United States increased to 70 thousand, and the number of new patients reached more than 80 thousand in 2018. The number of new cases and deaths increased annually in China. The incidence rate of bladder cancer was the first [3–6]. Clinically, it can be divided into transitional cell carcinoma, adenocarcinoma, squamous cell carcinoma, small cell carcinoma, metastatic carcinoma, and mixed types of cancer according to the tissue source of bladder cancer, among which transitional cell carcinoma is the most common [7–10].

Clinically, most patients with bladder cancer are NMIBC, and surgical treatment is the most effective and widely used treatment method [11–14]. NMIBC has the possibility of further developing into invasive bladder cancer. Therefore, the choice of surgical treatment for NMIBC aroused wide discussion and attention. A large number of researchers thought that radical cystectomy with radical cystectomy for NMIBC patients could significantly reduce the risk of recurrence of bladder cancer. However, great trauma was caused by this surgical method to the patient's body, and a variety of complications occurred in severe cases. In addition, the limitation of surgical indications was extremely strict, so its scope of clinical application was affected and could not be widely popularized [15, 16]. Iqbal et al. [17] investigated the incidence, risk factors, and survival outcomes associated with the pathologic rise from noninvasive to muscle-invasive bladder cancer after robot-assisted radical cystectomy. They found that patients with noninvasive bladder cancer who underwent surgical treatment had an increased incidence of muscle-invasive bladder cancer, which was associated with worse survival outcomes. Türk et al. [18] retrospectively analyzed the case data from 530 patients who underwent radical cystectomy or pelvic lymphadenectomy by selected surgeons between May 2005 and April 2016. They found that patients with early radical cystectomy had better disease-free survival and overall survival time than patients with pelvic lymphadenectomy. In recent years, transurethral resection of bladder tumors has appeared in the sight of researchers and doctors and has gradually developed into the main treatment method for patients with NMIBC [19, 20]. Transurethral resection of bladder tumors has many advantages, including less trauma, repeatable treatment, and rapid recovery. However, the risk of postoperative recurrence in patients with NMIBC after this operation was high [21–23].

Computed tomography (CT) is one of the most commonly used methods for the diagnosis of bladder cancer. Preoperative diagnosis can improve the accuracy of preoperative staging and detect the recurrence of bladder cancer after operation [24–26]. Conventional CT often uses two-dimensional slice observation, so many spatial data are lost, and the structural and morphological display of cancerous tissue is not complete and sufficient [27]. Imaging doctors cannot intuitively make accurate and objective judgments based on the observed images, which may lead to wrong diagnosis [28]. Three-dimensional images can completely, stereoscopically, and intuitively reproduce the tumor tissue morphology and structure. CT detection based on the three-dimensional reconstruction algorithm is helpful for clinicians to further observe and analyze, obtain more detailed information, and diagnose the disease more accurately and quickly [29].

To analyze the application value of CT images based on the three-dimensional reconstruction algorithm in perioperative nursing research and prognosis analysis of elderly patients with NMIBC, 124 patients with NMIBC were selected in this study. The patients were diagnosed by CT detection based on the three-dimensional reconstruction algorithm before operation. After the operation, the patients were divided into case group and control group for rapid comprehensive nursing and routine nursing. The recovery status of the two groups was analyzed and compared. In addition, the recurrence was detected by CT scanning, so as to evaluate the reference value of CT image information based on the three-dimensional reconstruction algorithm in preoperative diagnosis, postoperative nursing, and recurrence monitoring of NMIBC patients.

## 2. Materials and Methods

### 2.1. Research Object

A retrospective study was performed on 124 patients with NMIBC who underwent surgical treatment in the hospital from February 2, 2018, to June 2, 2020. The age of the patients was 55–75 years. They were divided into two groups, 62 in each group. All patients underwent transurethral resection of the bladder tumor. The patients in the case group received comprehensive nursing after the operation, and the patients in the control group took routine nursing measures. This study was approved by the medical ethics committee of the hospital, and all patients and their families signed informed consent.

Inclusion criteria were as follows: (1) patients with NMIBC diagnosed by imaging, CT, and pathology; (2) the patients who were in good condition without other serious organ diseases; (3) patients who cooperate with CT examination; (4) patients without any contraindications; and (5) the age range was 55–75 years.

Exclusion criteria were as follows: (1) patients with critical condition and survival less than half a year; (2) patients with other malignant tumors; (3) patients with mental illness who cannot be treated with surgery; and (4) patients whose family members did not consent and did not sign the informed consent.

### 2.2. Computed Tomography Imaging Examination

All patients underwent a CT imaging examination. The range between the bottom of the bladder and the ischial tubercle was included in the scanning position. Before scanning, the patient was instructed by the doctor to drink a large amount of water to keep the bladder in a full state. First, the plain scanning mode was performed, and iohexol (300 mg/mL) was injected at a uniform speed. The patients were scanned in enhanced mode after 45 s, and the delayed scan was completed after 5 min.

### 2.3. Three-Dimensional Reconstruction Algorithm

In this study, the improved marching cubes (MC) algorithm was used to reconstruct three-dimensional images. Multiple contour lines were set for all CT slices and were named *L*1, *L*2,…, *Ln*. Each voxel (*a*, *b*, *c*) in the data was assigned to the function *f* (*a*, *b*, *c*). When (*a*, *b*, *c*) was outside all contour lines, it was expressed as

(1) $$\begin{array}{c} f\left(a,\;b,c\right)=-1. \end{array}$$

When (*a*, *b*, *c*) was above any contour line, it was expressed as

(2) $$\begin{array}{c} f\left(a,\;b,c\right)=0. \end{array}$$

When (*a*, *b*, *c*) was within any contour line, it was expressed as the following equation:

(3) $$\begin{array}{c} f\left(a,\;b,c\right)=1. \end{array}$$

Each point may have a result of 0, −1, or 1. When the edge interface passed through the vertex whose function *f* (*a*, *b*, *c*) was 0 and if the values of two vertex functions *f* (*a*, *b*, *c*) located on an edge were different signs, the edge interface would intersect with the edge. If the values of two vertex functions *f* (*a*, *b*, *c*) located on an edge were different signs, the edge interface would not intersect with the edge. When an edge interface intersected with an edge, the midpoint of the edge was usually taken as the intersection point, and different intersection points were connected in order to obtain the reconstructed surface. The function *f* (*a*, *b*, *c*) of each vertex would have three cases: 0, −1, and 1. In addition, the normal direction of the vertex could be calculated by the central difference method, and the state value of the vertex could be displayed according to the function *f* (*a*, *b*, *c*). Then, the normal direction is shown as follows:

(4) $$\begin{array}{c} M_{a}=\frac{f\left(a-1,b,c\right)-f\left(a+1,b,c\right)}{2},\\ M_{a}=\frac{f\left(a,b-1,c\right)-f\left(a,b+1,c\right)}{2},\\ M_{a}=\frac{f\left(a,b,c-1\right)-f\left(a,b,c+1\right)}{2}. \end{array}$$

The triangular surface generated after three-dimensional reconstruction needed to be simplified by the deletion algorithm so as to improve the speed of model reconstruction. The priority function was expressed as *Y*, as shown in the following equation:

(5) $$\begin{array}{c} Y\left(s\right)=C_{t}T\left(s\right)+C_{x}X\left(s\right)+C_{g}G\left(s\right). \end{array}$$

In equation (5), *s* was the edge to be processed, and the flatness of the triangle connected with *s* was expressed as *T* (*s*). The normal direction of this kind of triangle could be expressed as

(6) $$\begin{array}{c} {\dot{L}}_{i}\left(i=1,2,\ldots \ldots ,n\right). \end{array}$$

Then,

(7) $$\begin{array}{c} T\left(s\right)=Max\left(1-{\dot{L}}_{i}\;{\dot{L}}_{j}\right). \end{array}$$

In the equation (7), *G* (*s*) was the length of one side *s* and *X* (*s*) was the shape coefficient of the triangle with side *s* connected.

### 2.4. Surgical Treatment

All patients with NMIBC were given general anesthesia. Transurethral resection of the bladder tumor was performed at the bladder lithotomy site. Different parameters of the resection mirror were set. The electrocoagulation power and resection power were 60–80 W and 80 W, respectively. The resection range was 1 cm away from the edge of the tumor base to ensure complete resection of the tumor base. During the operation, the superficial muscle layer or the whole layer of the bladder wall could be selected according to the specific situation. When the tumor was too large, the protrusion tissue was first removed, then the tumor base was completely removed, and electrocautery was used to stop bleeding.

### 2.5. Postoperative Nursing Process

After the operation, the patients in the case group and the control group were treated with comprehensive nursing and routine nursing. Routine nursing: electrocardiographic (ECG) monitoring was performed 24 hours after the operation to observe the changes in blood pressure, respiration, pulse, and other parameters. Comprehensive nursing intervention in the case group: on the basis of routine nursing, psychological health counseling was conducted. Besides, timely communicating with patients and their families, popularizing medical-related knowledge, and instructing the significance of postoperative bladder flushing should be conducted, so as to alleviate the tension of patients and make patients cooperate with treatment in a good emotional state. Nursing care of bladder flushing: attention should be paid to the flushing operation, and the changes in flushing fluid should be timely monitored. Nurses and family members should timely react with doctors. The temperature, dosage, and flushing speed of flushing fluid were controlled as required. Nursing of drainage tube: the drainage tube was properly fixed to ensure its patency in the whole process, bladder spasm was prevented, the change of drainage fluid was monitored in real time, and the drainage speed was controlled. Nurses and family members should timely communicate with doctors for adjustment in time.

### 2.6. Observation and Evaluation Indicators

The general basic data of the two groups were collected, analyzed, and compared, including average age, proportion of men and women, course of disease, average tumor diameter, and proportion of patients with single and multiple tumors.

Based on the pathological examination results, three common index CT images based on the three-dimensional reconstruction algorithm were selected to evaluate the preoperative diagnostic effect of NMIBC patients, namely, accuracy, specificity, and sensitivity. The calculation methods are shown in the following equations:

(8) $$\begin{array}{c} \text{accuracy }=\;\frac{A\;+\;B}{A\;+\;C\;+\;B\;+\;D},\\ \text{specificity }=\;\frac{B}{C\;+\;B},\\ \text{sensitivity }=\;\frac{A}{D\;+\;A}. \end{array}$$

In the above equation, *A* was true positive, indicating that the diagnostic result was positive and actually positive; *B* meant true negative, indicating that the diagnosis result was negative and actually negative; *C* was false positive, meaning that the diagnostic result was positive and actually negative; *D* was false negative, indicating that the actual result was positive and the diagnostic result was negative.

A receiver operating characteristic (ROC) curve was used to represent the diagnostic ability of CT information for patients with NMIBC, and the area under the curve (AUC) was determined according to ROC.

A self-rating anxiety scale (SAS) [30] was used to evaluate the psychological status of the two groups. The total score was 100. The higher the score was, the more serious the anxiety state was. The frequency of bladder spasm, bladder flushing time, and indwelling time of the drainage tube were recorded and compared between the two groups. The changes of tumor markers of bladder cancer specific antigen-1 (BLCA-1) and cyto-keratin 19 fragment antigen 21-1 (CYFRA21-1) were recorded in two groups of patients after operation. The quality of life of patients at 6 months after operation was evaluated by using the European Cancer Research and Treatment Organization quality of life core questionnaire. The scores were determined by five aspects: role, body, emotion, social, and cognitive function. The higher the score was, the better the quality of life of patients after operation was. The postoperative complications of the two groups were recorded and compared, and the complications such as electroresection syndrome, urinary tract infection, and massive hemorrhage were observed and analyzed. One year after the operation, CT image scanning based on the three-dimensional reconstruction algorithm was performed to check the recurrence of the two groups.

### 2.7. Statistical Methods

SPSS software was used to analyze the data. The data conforming to normal distribution was expressed by mean ± *s*, and the measurement data was expressed by *t*-test, chi-square test, (*χ*2) was used to indicate the counting data, and *P* < 0.05 indicated that there was a statistical difference.

## 3. Results

### 3.1. Comparison Results of Basic Conditions of Patients

The basic conditions of the two groups were recorded and compared. It was found that there was no significant difference between the case group and the control group in terms of average age, proportion of male patients, average tumor diameter, duration of disease, and number distribution of patients with multiple tumors (*P* < 0.05). In addition, there was no significant difference between the two groups in the proportion of patients with hematuria, frequent urination, urgent urination, dysuria, and obvious weight loss (*P* < 0.05). The specific results are illustrated in Figures 1 and 2.

### 3.2. Computed Tomography Imaging Results of Patients

Figure 3 shows the CT image of a 57-year-old male. There were multiple multicolor lumps on the left lateral wall and left posterior wall of the bladder. The largest one was located 2.5 cm above the left ureter, with a wide base. There was necrosis on the tumor surface, and the rest of the bladder mucosa was smooth.

Figure 4 shows the CT image of a 63-year-old male. There was a papillary mass on the left posterior wall of the bladder, with 3 × 3 cm in size and a broad base close to the right ureteral opening. The vascular pedicle was clear.

### 3.3. Diagnostic Ability of Computed Tomography Images

By calculating the accuracy, specificity, and sensitivity, it was found that the accuracy, specificity, and sensitivity of CT imaging information based on the three-dimensional reconstruction algorithm in diagnosing NMIBC patients were 89.38, 93.77, and 84.39, respectively. The specific results are revealed in Figure 5.

The ROC curve was drawn according to the specificity and sensitivity of CT imaging information in diagnosing NMIBC patients, as shown in Figure 6. In addition, the AUC was determined to be 0.871 according to the ROC.

### 3.4. SAS Score Results of Two Groups

After treatment, the SAS scores of the two groups were measured. The results showed that the scores of the case group were significantly lower than those of the control group (*P* < 0.05). The specific results are shown in Figure 7.

### 3.5. Comparison of the Incidence of Bladder Spasm, Bladder Flushing, and Indwelling Time of Drainage Tube between the Two Groups

The incidence of bladder spasm, bladder flushing, and indwelling time of the drainage tube in the two groups were recorded and compared. The results indicated that the incidence of bladder spasm (9.68%), bladder flushing time (1.56 d), and retention of drainage tube time (2.68 d) in the case group were obviously lower compared to the control group (30.65%, 2.32 d, and 5.19 d) (*P* < 0.05). The specific results are shown in Figure 8.

### 3.6. Comparison of Tumor Markers between the Two Groups

The levels of tumor markers after operation in the two groups were recorded and compared. The results showed that serum BLCA-1 (3.72 ng/mL) and CYFRA21-1 (5.68 *μ*g/mL) in the case group were signally lower than those in the control group, with a statistically considerable difference (*P* < 0.05).  Figure 9 illustrates the specific results.

### 3.7. Comparison of Quality of Life Scores between the Two Groups

The postoperative quality of life indexes of the two groups were recorded and compared. The results showed that, in contrast to the control group, the scores of role function (89.82 points), emotional function (84.76 points), somatic function (79.23 points), and social function (73.93 points) in the case group were markedly higher (*P* < 0.05). The specific results are shown in Figure 10.

### 3.8. Comparison of Postoperative Complications and Recurrence Rate between the Two Groups

The postoperative complications of the two groups were recorded and compared. The results showed that compared with the control group, the number of patients with postoperative urinary tract infection and electroresection syndrome in the case group was significantly lower (*P* < 0.05), and there was no urethral stricture in the two groups. In addition, one year after the operation, CT examination showed that the recurrence rate in the case group (6.45%) was significantly lower than that in the control group (22.58%) (*P* < 0.05).  Figure 11 suggests the specific results.

## 4. Discussion

At present, the incidence rate and mortality rate of bladder cancer are increasing, and it has the characteristics of high malignancy and poor prognosis. It has seriously damaged the physical and mental health of patients. In men, bladder cancer has been ranked fifth in cancer mortality rate, and in women, it has been ranked in the top ten. Therefore, timely diagnosis and effective treatment of bladder cancer are particularly important [31]. About 70% of the clinical patients are NMIBC patients, but non-muscle-invasive bladder cancer patients also have a higher risk of metastasis. Surgical treatment is the main means of clinical treatment for bladder cancer. Preoperative diagnosis of bladder tumor by CT is very important for determining the stage, location, and size of the bladder tumor. CT is one of the common methods for the clinical diagnosis of bladder cancer. Preoperative diagnosis can improve the accuracy of preoperative staging and can detect the recurrence of bladder cancer. CT detection based on a three-dimensional reconstruction algorithm is helpful for clinicians to further observe and analyze, obtain more deep information, and confirm the operation plan more accurately and quickly [32]. To analyze the application value of CT image based on three-dimensional reconstruction algorithm in perioperative nursing research and prognosis analysis of elderly patients with NMIBC in urology, 124 patients with NMIBC were selected and divided into case group and control group. Before operation, CT detection based on the three-dimensional reconstruction algorithm was used to diagnose the tumor. The results showed that there was no significant difference in the average age, the proportion of male patients, the average tumor diameter, the length of disease course, and the number distribution of patients with multiple tumors (*P* < 0.05). In addition, there was no significant difference between the two groups in the proportion of patients with hematuria, frequent urination, urgent urination, dysuria, and obvious weight loss (*P* < 0.05), which showed that the basic conditions of the two groups were the same and increased the comparability of follow-up parameters. By calculating the accuracy, specificity, and sensitivity, it was found that the accuracy, specificity, and sensitivity of CT imaging information based on the three-dimensional reconstruction algorithm in diagnosing NMIBC patients were 89.38, 93.77, and 84.39, respectively. The ROC curve was drawn according to the specificity and sensitivity of CT imaging information in diagnosing NMIBC patients, and the AUC was determined to be 0.871 according to ROC. This indicated that the CT image based on the three-dimensional reconstruction algorithm had a strong diagnostic ability for NMIBC patients. The results of comparative analysis of the two diagnostic methods of CT and pathology in multiple bladder cancer pathologies showed that the coincidence rate between CT diagnosis and pathological diagnosis was high. It could provide a reference for the clinical diagnosis of MNIBC patients, which was more consistent with the results of this study [33].

In this study, the patients were divided into case group and control group for rapid comprehensive nursing and routine nursing. The recovery status of the two groups was analyzed and compared. The recurrence was detected by CT scanning, so as to evaluate the reference value of CT image information based on the three-dimensional reconstruction algorithm in preoperative diagnosis, postoperative nursing, and recurrence monitoring of NMIBC patients. The results showed that after surgical treatment and nursing, compared with the control group, the SAS score in the case group was significantly lower (*P* < 0.05). The incidence of bladder spasm in the case group was significantly lower, the bladder flushing and drainage tube retention time were significantly shorter (*P* < 0.05), and the tumor markers BLCA-1 and CYFRA21-1 in the serum of the case group were significantly lower (*P* < 0.05). The scores of emotional function, physical function, and social function increased significantly (*P* < 0.05), and there was no significant difference in cognitive function between the two groups (*P* > 0.05). Compared with the control group, the number of patients with postoperative urinary tract infection and electroresection syndrome in the case group decreased significantly (*P* < 0.05). There was no urethral stricture in both groups. In addition, one year after the operation, CT examination showed that the recurrence rate of patients in the case group was significantly lower than that in the control group (*P* < 0.05), indicating that postoperative comprehensive nursing was particularly important for patients with NMIBC. CT detection could play a great role in the postoperative detection and prognosis evaluation of NMIBC. In some studies, the recurrence rate of patients with NMIBC decreased significantly after surgical treatment and one year after comprehensive nursing, which was consistent with the results of this study [34]. In conclusion, CT detection based on a three-dimensional reconstruction algorithm was particularly important for preoperative diagnosis, prognosis, and recurrence monitoring of NMIBC patients.

## 5. Conclusion

124 patients with NMIBC received CT examination based on the three-dimensional reconstruction algorithm and received rapid comprehensive care and conventional care. The results showed that CT images based on the three-dimensional reconstruction algorithm had a strong diagnostic ability for NMIBC patients, and postoperative comprehensive care was particularly crucial for NMIBC patients. Besides, CT detection could play a huge role in postoperative detection and prognosis assessment of NMIBC. Postoperative comprehensive nursing could not only shorten the bladder flushing and retention of drainage tube time of NMIBC patients but also reduce the postoperative recurrence rate and improve the prognosis. The deficiency of this study was that the sample size of the research object had a single source and did not have randomness and wide applicability. In the future research, multilocation and multitype sample size analysis and research will be considered, so as to provide a more practical and effective reference for CT imaging examination and its monitoring in preoperative diagnosis, prediction, and recurrence of NMIBC patients.

## Figures and Tables

**Figure 1:** Comparison results of basic conditions of two groups of patients. (a) The comparison of average age and the male ratio between the two groups; (b) the comparison of average tumor diameter and course of disease between the two groups; (c) the comparison of the number of patients with multiple and single tumors between the two groups.

**Figure 2:** Comparison of clinical symptoms between the two groups. (a) The comparison of the number of patients with hematuria, frequent urination, and urgent urination in the two groups; (b) the comparison of the number of patients with dysuria and significant weight loss in the two groups.

**Figure 3:** The CT image of a 57-year-old male patient, with a history of high blood pressure.

**Figure 4:** The CT image of a 63-year-old male patient. The general condition was good, and he was admitted after 8 days of hematuria.

**Figure 5:** Evaluation of the ability of CT imaging information to diagnose NMIBC patients.

**Figure 6:** ROC curve results of NMIBC patients diagnosed by CT imaging information.

**Figure 7:** Comparison of SAS scores between the two groups. *∗* indicates significant difference, *P* < 0.05.

**Figure 8:** Comparison of the incidence of bladder spasm, bladder flushing, and indwelling time of drainage tube between the two groups. (a) The comparison of the incidence of bladder spasm between the two groups; (b) the comparison of bladder flushing time between the two groups; (c) the comparison of the retention time of the bladder drainage tube between the two groups. *∗* indicates a significant difference: *P* < 0.05.

**Figure 9:** Comparison of tumor markers in serum between the two groups. *∗* indicates significant difference, *P* < 0.05.

**Figure 10:** Quality of life score results of two groups of patients. *∗* indicates significant difference, *P* < 0.05.

**Figure 11:** Comparison of postoperative complications and recurrence between the two groups. (a) The comparison results of complications between the two groups; (b) the comparison results of postoperative recurrence between the two groups. *∗* indicates significant difference, *P* < 0.05.

## Data Availability

The data used to support the findings of this study are available from the corresponding author upon request.
